The article "Reconstruction Algorithm-Based CT Imaging for the Diagnosis of Hepatic Ascites" was published in 2022. Journal: Comput Math Methods Med.

# Reconstruction Algorithm-Based CT Imaging for the Diagnosis of Hepatic Ascites

**DOI:** 10.1155/2022/1809186

**Published:** 2022-05-04

**Authors:** Huitao Zhang, Wenhao Lv, Haofeng Diao, Li Shang

**Affiliations:** ^1^Department of Gastroenterology, The No.4 People's Hospital of Hengshui City, Hengshui 053000, China; ^2^Department of Spine Surgery, The No.4 People's Hospital of Hengshui City, Hengshui 053000, China

## Abstract

The study was aimed at exploring the diagnostic value of artificial intelligence reconstruction algorithm combined with CT image parameters on hepatic ascites, expected to provide a reference for the etiological evaluation of clinical abdominal effusion. Specifically, the adaptive iterative hard threshold (AIHT) algorithm for CT image reconstruction was proposed. Then, 100 patients with peritoneal effusion were selected as the research subjects. After 8 cases were excluded, the remaining was divided into 50 cases of the S1 group (hepatic ascites) and 42 cases of the D0 group (cancerous peritoneal effusion). Gemstone energy spectrum CT scanning was performed on all patients, and CT image parameters of the two groups were compared. It was found that CT value of mixed energy, CT value of 60-100 KeV single energy, concentration value of water (calcium), concentration value of water (iodine), and slope of energy spectrum curve in the S1 group were significantly lower than those in the D0 group (*P* < 0.05). The effective atomic number in the S1 group was significantly higher than that in the D0 group (*P* < 0.05). Of the 50 patients in the S1 group, 3 (6%) had an ascending and 47 (94%) had a descending spectral curve. Of the 42 patients in the D0 group, 37 (88.1%) had an ascending and 5 (11.9%) had a descending spectral curve. The sensitivity and specificity of water (iodine) were 0.927 and 0.836, respectively. The sensitivity and specificity of water (calcium) were 0.863 and 0.887, respectively. For different scan ranges ([0,90]; [0,120]), root mean square error (RMSE) of AIHT reconstructed image was significantly smaller than that of traditional algorithm, while peak signal-to-noise ratio (PSNR) was opposite. The differences were statistically significant (*P* < 0.05). In conclusion, AIHT-based CT images can better display the distribution of hepatic ascites, and the parameters of CT value, effective atomic number, water (iodine), water (calcium), and spectral curve can all provide help for the identification of hepatic ascites. Especially, water (iodine) and water (calcium) demonstrated high diagnostic performance of hepatic ascites.

## 1. Introduction

Hepatic ascites refers to ascites caused by liver function damage and portal hypertension due to cirrhosis. It is one of the most common complications of cirrhosis [1–3]. In the natural course of chronic liver disease, ascites is an important sign that cirrhosis progresses to decompensation of liver function [4–6]. The clinical symptoms are mainly abdominal distension, abdominal distension, and mild abdominal pain, and symptoms such as dyspnea, nausea, vomiting, loss of appetite, satiety, and edema of lower limbs may occur [7, 8]. The increasing ascites in the liver will affect people's appetite and easily lead to abdominal distension and poor breathing. In severe cases, it will affect the kidney to generate urine [9]. When the liver ascites develops to the middle and late stage, it will affect the gastrointestinal function, manifesting as abdominal pain, abnormal stool, and black stool [10]. There is no exact number for the life span of patients with hepatic ascites. If some patients are treated regularly in time, the patients can effectively recover [11].

At present, there are X-ray, ultrasound, magnetic resonance imaging (MRI), and computed tomography (CT) for the clinical diagnosis of ascites. X-ray and ultrasound have poor diagnostic effect on ascites and cannot make a definite diagnosis [12]. Although ordinary CT can detect the occurrence of ascites with high resolution, it cannot judge the nature of ascites. MRI can distinguish purulent, blood, even benign, and malignant effusion to a certain extent by combining various signals, but it has some disadvantages such as high price, slow imaging speed, and many taboos [13, 14]. Gem energy spectrum imaging is a rare platform for low-dose energy spectrum imaging, and energy spectrum imaging has been realized by high- and low-pressure instantaneous X-ray emission system and ultrafast gem energy spectrum detector [15]. Doctors can use energy spectrum imaging to analyze the chemical composition of human body and make more accurate pathological diagnosis, which can provide more reliable information for the evaluation of the nature of ascites [16]. When CT is used to diagnose the thoracic cavity, the projection data can only be collected within a limited rotation angle, so it has the problem of incomplete data. Ahn et al. [17] reconstructed CT images by filtering back projection (FBP), hybrid iterative reconstruction (HIR), and iterative model reconstruction (IMR) algorithms. Different reconstruction algorithms were found to affect the histogram and texture features, and reconstruction algorithms showed a stronger effect in focal liver disease than in liver parenchyma or renal cyst. Song et al. [18] enrolled 75 patients with primary abdominal malignancy and reconstructed liver CT images at portal stage using filtered post projection (FBP) or HIR algorithm with six different iterative reconstruction intensities. It was found that HIR algorithm can reduce image noise and provide better image quality than FBP. Traditional filtered back projection (FBP) reconstruction algorithm will lead to obvious landslide artifacts in reconstructed images, which will affect the results of nondestructive testing and medical diagnosis. Therefore, it is necessary to propose a more accurate CT image reconstruction algorithm.

To sum up, the causes of ascites are complex and varied, and how to identify hepatic ascites quickly and accurately is an important topic in current research. Therefore, 100 patients diagnosed with peritoneal effusion were included in this study, and gem energy spectrum CT scan under iterative reconstruction algorithm was performed, so as to explore the evaluation value of the iterative reconstruction algorithm combined with CT images for peritoneal effusion in cirrhosis.

## 2. Materials and Methods

### 2.1. Research Subjects

In this study, 100 patients with peritoneal effusion diagnosed in hospital from May 1, 2016, to October 1, 2019, were selected as the research subjects. Among them, 8 cases were excluded due to the low amount of peritoneal effusion, which could not provide enough effusion layer to circle sufficient areas of interest, and 92 cases left. Then, according to the clinical diagnosis results, the patients were divided into 50 hepatic ascites group (S1) and 42 D0 group (carcinomatous peritoneal effusion group). This study had been approved by ethics committee of hospital, and patients and their families were informed of this study and had signed the informed consent form.

Inclusion criteria for group S1: (I) patients with cirrhosis confirmed by liver biopsy; (II) the patient was not complicated by malignant tumor; (III) laboratory tests proved that the abdominal effusion was benign; (IV) no contraindications for abdominal puncture; and (V) patients without contraindications for CT examination.

Inclusion criteria for group D0: (I) cytological examination showed cancer cells; (II) laboratory tests proved that the abdominal effusion was cancerous; (III) biopsy of focal tissue proved that the placeholder was cancerous; (IV) no contraindications for abdominal puncture; and (V) patients without contraindications for CT examination.

Exclusion criteria: (I) low amount of abdominal fluid; (II) patients with tuberculosis, renal failure, and heart failure; (III) patients with cirrhosis and malignant tumors; (IV) patients with low level of cultural knowledge, difficulty in communication, and excessive anxiety; (V) poor inspection compliance; and (VI) CT image quality was poor, with large motion artifacts or metal artifacts.

### 2.2. CT Examination Methods

Before the examination, the patient was told to drink 1000 mL water 10 minutes before the examination. The patient was in a supine position with hands raised above the head. CT equipment was used to scan from the parietal layer to the pubic symphysis layer. Scanning parameters are as follows: frame rotation speed of 0.5 seconds/r, pitch 0.975, tube voltage switching between 140 kVP and 80 kVP, tube current 450 mA, layer thickness 4.5 mm, layer spacing 4.5 mm, field of vision 450 mm, and collimator 50 mm.

The obtained images were transmitted to the workstation for processing. Through the image of 100 KeV mixed energy, the average CT value of mixed energy was obtained. The following data were obtained through the image of 50 KeV single energy: (I) average value of different base substance pairs: water (iodine) concentration and water (calcium) concentration; (II) CT values at each single energy of 30-100 KeV; (III) average value of effective atomic number; and (IV) the slope of energy spectrum attenuation curves of cirrhotic and cancerous peritoneal effusion.

### 2.3. AIHT Image Reconstruction Algorithm

In finite angle CT reconstruction, it is difficult to select the parameters of regularized image reconstruction algorithm based on optimization theory, which is generally selected by experience. Therefore, it is necessary to adjust parameters repeatedly to achieve better reconstructed image quality, which greatly increases the time cost [19]. In the study, the l-shaped curve strategy is introduced and a reconstruction algorithm with adaptive selection of hard threshold parameters is proposed, so that the reconstruction process of finite angle CT can be intelligently realized.

Firstly, the algorithm model is proposed based on regularization terms.

(1) $$\begin{array}{c} \underset{h\in \Omega }{\arg\min}\left\{\frac{{\left\|Zh-l^{\vartheta }\right\|}_{B}^{2}}{2}+\underset{i}{\sum }\beta_{i}{\left\|\left({Ah}_{2}\right)\right\|}_{\tau }\right\}, \end{array}$$

where *Z* represents the matrix of finite angle CT and ‖.‖_*B*_ represents the weighted norm, *B* represents the diagonal matrix, *l* represents the initial image, *l*^*ϑ*^ represents the projected data of noise level *ϑ*, *β*_*i*_ represents the regularization parameter, ‖.‖_*τ*_ represents the nonzero number, *A* represents the fragment constant, and *B* is the spline wavelet compact frame. Then, the corresponding filter can be expressed as follows.

(2) $$\begin{array}{c} k_{0}=\frac{\left[1,2,1\right]}{2*2},\\ k_{1}=\frac{\sqrt{2}\cdot \left[1,0,‐1\right]}{2*2},\\ k_{2}=\frac{\left[‐1,2,1\right]}{2*2}, \end{array}$$

where *k* represents the filter parameter. The simultaneous algebra reconstruction technique (SART) is used, and iterative techniques can be performed without storing system matrices. So, the SART algorithm is introduced to solve the model, and the iteration form can be expressed as follows.

(3) $$\begin{array}{c} h^{\left(\text{m}\right)}*=h^{\left(\text{m}\right)}-\frac{V^{‐1}Z^{G}B\left({Zh}^{\left(\text{m}\right)}‐l^{\vartheta }\right)}{g}, \end{array}$$

where *Z* represents a diagonal matrix. Considering that the regularization term is in the wavelet domain, while the iteration domain is in the image domain, the wavelet transform is needed to transform the image into the wavelet domain. Then, the equation below is obtained.

(4) $$\begin{array}{c} \underset{h\in \Omega }{\arg\min}\left\{\frac{g{\left\|Ah-{Ah}^{\left(\text{m}\right)}*\right\|}_{2}^{2}}{2}+\underset{i}{\sum }\beta_{i}{\left\|{\left(Ah\right)}_{\text{i}}\right\|}_{\tau }\right\}. \end{array}$$

Components can be expressed as follows.

(5) $$\begin{array}{c} \underset{h}{\arg\min}\left\{\frac{g\sum_{i}{\left\|Ah-{Ah}^{\left(\text{m}\right)}*\right\|}_{2}^{2}}{2}+\underset{i}{\sum }\beta_{i}{\left\|{\left(Ah\right)}_{\text{i}}\right\|}_{\tau }\right\}. \end{array}$$

Through equation (5), the equation below is obtained.

(6) $$\begin{array}{c} {\left({Ah}^{\left(\text{m}+1\right)}\right)}_{i}\in F_{\beta i}\left({\left({Ah}^{\left(\text{m}\right)}*\right)}_{\text{i}}\right), \end{array}$$

where *β*_*i*_^∗^ is the hard threshold and $\beta_{i}^{*}=\sqrt{2\beta_{i}/g}$. *F*_*β*_*i*_^∗^_(.) is a function, and

(7) $$\begin{array}{c} F_{\beta_{i}^{*}}\left(y_{i}\right)=\left\{\begin{array}{cc} 0 & \left|y_{i}\right|<\beta_{i}^{*},\\ 0,y_{i} & \left|y_{i}\right|=\beta_{i}^{*},\\ y_{i} & \left|y_{i}\right|>\beta_{i}^{*}. \end{array}\right. \end{array}$$

The wavelet coefficient can be obtained by transforming the form of equation (6).

(8) $$\begin{array}{c} {Ah}^{\left(\text{m}+1\right)}\in F_{\beta *}\left({Ah}^{\left(\text{m}\right)}*\right). \end{array}$$

Further wavelet framework reconstruction can obtain the equation below.

(9) $$\begin{array}{c} h^{\left(\text{m}+1\right)}\in Z^{G}F_{\beta *}\left({Ah}^{\left(\text{m}\right)}*\right). \end{array}$$

The algorithm in this study can be divided into three steps: SART algorithm solving, wavelet compact frame transformation, and hard threshold solving, set as AIHT.

### 2.4. Quality Assessment of Reconstructed CT Images

In this study, root mean square error (RMSE) and peak signal-to-noise ratio (PSNR) were used to evaluate the quality of the reconstructed CT image, expressed as follows.

(10) $$\begin{array}{c} \text{RMSE}=\sqrt{\frac{\sum_{i=1}^{M}{\left(P_{i}-Q_{i}\right)}^{2}}{M}},\\ \text{PSNR}=10\log_{10}\frac{{\left\|Q\right\|}_{\infty }^{2}}{{\text{RMSE}}^{2}}, \end{array}$$

where *P* represents reconstructed image, *Q* represents the original image, and *M* represents window size.

Different scan ranges ([0,90]; [0,120]) are selected as experimental samples, and the finite angle CT reconstruction algorithm based on multiplicative regularization (MR) and finite angle CT iterative reconstruction algorithm based on wavelet frame (WF) are introduced and compared with AIHT algorithm in this study.

### 2.5. Statistical Methods

SPSS19.0 statistical software was used for data processing in this study. Mean ± standard deviation ($\overset{¯}{x}\pm s$) was used for measurement data, and percentage (%) was used for count data. Pairwise comparison was performed by one-way ANOVA. The difference was statistically significant at *P* < 0.05.

## 3. Results

### 3.1. Reconstruction Performance Comparison of Algorithms

As shown in Figure 1(a), in CT image within the scanning range of [0,90], the RMSE index of reconstructed images by AIHT algorithm was significantly lower than that by MR algorithm and WF algorithm, and the difference was statistically significant (*P* < 0.05); the PSNR index of AIHT algorithm was significantly higher than that of MR algorithm and WF algorithm, and the difference was statistically significant (*P* < 0.05).  Figure 1(b) shows the image reconstructed by the algorithm. It was noted that the overall quality of the image reconstructed by AIHT algorithm was better than that of MR algorithm and WF algorithm, which effectively improved the degradation of boundary structure information caused by the discomfort of finite angle CT reconstruction.

As shown in Figure 2(a), in CT image within the scanning range of [0,120], the RMSE index of reconstructed images by AIHT algorithm was significantly lower than that by MR algorithm and WF algorithm, and the difference was statistically significant (*P* < 0.05); the PSNR index of AIHT algorithm was significantly higher than that of MR algorithm and WF algorithm, and the difference was statistically significant (*P* < 0.05).  Figure 2(b) shows the image reconstructed by the algorithm. It was noted that the overall quality of the image reconstructed by AIHT algorithm was better than that of MR algorithm and WF algorithm, and the degradation of the boundary structure information of the reconstructed image was significantly improved.

### 3.2. Comparison of General Data between the Two Groups

As shown in Figure 3, there were no significant differences in age, male and female ratio, course of disease, body mass index (BMI), diabetes, hypertension, and smoking between the two groups (*P* > 0.05).

### 3.3. CT Image Data of some Patients

As shown in Figure 4, diffuse or nonuniform decrease in liver parenchyma density (decreased CT value) was observed on plain and enhanced CT scan, liver contour was uneven, and liver fissure was widened. The volume of left lobe and caudate lobe increased, and the volume of right lobe decreased.

Postoperative changes in Figure 5 are as follows: increased abdominal and pelvic effusion, abdominal intestinal wall edema and thickening, multiple small lymph nodes in the mesentery, bilateral renal cysts, and calcification of the prostate.

### 3.4. Comparison of CT Values between the Two Groups

Figure 6 shows the CT values of patients in the two groups under mixed energy and single energy. It was noted that the CT value of mixed energy in the S1 group was significantly lower than that in the D0 group, and the difference was statistically significant (*P* < 0.05). There was no statistically significant difference in the single-energy CT value of KeV between the S1 group (30-50) and D0 group (*P* < 0.05). The single-energy CT value of KeV in the S1 group (60-100) was significantly lower than that in the D0 group, and the difference was statistically significant (*P* < 0.05).

### 3.5. Comparison of Paired Base Substance Concentration and Effective Atomic Number between the Two Groups

Figure 7 shows the concentration of paired basal substances and effective atomic number between the two groups. It was noted that the concentration values of water (calcium) and water (iodine) in the S1 group were significantly lower than those in the D0 group, and the differences were statistically significant (*P* < 0.05). The effective atomic number in the S1 group was significantly higher than that in the D0 group, and the difference was statistically significant (*P* < 0.05).

### 3.6. Spectral Curve Analysis Results of the Two Groups

According to Figure 8(a), the slope of spectral curve in the S1 group was significantly lower than that in the D0 group, and the difference was statistically significant (*P* < 0.05).

According to the comparison of different types of spectral curves (Figures 8(b) and 8(c)), 3 cases (6%) and 47 cases (94%) of the 50 patients in the S1 group had an upward and downward spectral curve; of the 42 patients in the D0 group, 37 patients (88.1%) had an ascending spectral curve, and 5 patients (11.9%) had a descending spectral curve.

### 3.7. Diagnostic Efficacy of Some Parameters of CT Images on Hepatic Ascites

Figure 9 shows the diagnostic efficacy of some parameters of CT image on hepatic ascites. It was noted that the sensitivity and specificity of water (iodine) and water (calcium) were good in the diagnosis of hepatic ascites. The sensitivity and specificity of water (iodine) were 0.927 and 0.836, respectively. The sensitivity and specificity of water (calcium) were 0.863 and 0.887, respectively. The spectral curve slope had the lowest sensitivity and specificity in the diagnosis of hepatic ascites, which were 0.815 and 0.788, respectively.

## 4. Discussion

Peritoneal effusion is the pathological accumulation of body fluid in the peritoneal cavity. Under normal circumstances, the peritoneal cavity contains a small amount of fluid which can play a lubricating role between the visceral and wall layers of the peritoneum [20]. In a pathological condition, the amount of the liquid will increase. Peritoneal effusion is just a clinical symptom, rather than an independent disease. Its etiology is varied, such as cirrhosis of the liver decompensation period, malignant placeholder lesions, and tuberculous peritonitis, so to find the right way to evaluate liver cirrhosis ascites is necessary [21, 22]. Gem CT can help doctors to make early and differential diagnosis of diseases and also be helpful for the diagnosis of ascites. Therefore, the AIHT image reconstruction algorithm was proposed in this study, and its performance is compared with that of previous algorithms. The results showed that, in different scan ranges of [0,90] and [0,120], the RMSE index of AIHT algorithm was significantly lower than that of MR algorithm and WF algorithm, while the PSNR index was significantly higher than that of MR algorithm and WF algorithm (*P* < 0.05), which indicated that AIHT algorithm proposed in this study had a good effect on CT image reconstruction. The boundary structure information degradation caused by inappropriate finite angle CT reconstruction was improved effectively.

Then, 100 patients diagnosed with peritoneal effusion in hospital were selected as the research subjects, and 8 cases were excluded. The remaining was divided into 50 cases of the S1 group (hepatic ascites) and 42 cases of the D0 group (cancerous peritoneal effusion). All of them were scanned by GE Discovery 750 gemstone energy spectrum CT, and the CT image parameters of the two groups were analyzed. It was found that there was no statistically significant difference in KeV single-energy CT values between the S1 group (30-50) and D0 group (*P* < 0.05), which was different from previous studies, possibly due to the weak X-ray penetration at low energy level, which resulted in fewer X-ray particles involved in imaging and increased image noise [23]. However, the CT values of mixed energy and 60-100 KeV single-energy CT values in the S1 group were significantly lower than those in the D0 group, and the differences were statistically significant (*P* < 0.05), indicating that there are significant differences in the composition and density of hepatic ascites and cancerous peritoneal effusion. As for the concentration of paired base substances, the concentration values of water (calcium) and water (iodine) in the S1 group were significantly lower than those in the D0 group, and the differences were statistically significant (*P* < 0.05). Gem energy spectrum CT obtained dual-energy data through instantaneous high and low energy switching and changed the absorption projection of space into the density projection of material to realize substance separation. The results were related to the different types of hepatic ascites and cancerous peritoneal effusion [24]. Effective atomic number means that the atomic number of an element is the same as the X-ray absorption attenuation coefficient of a substance, and the atomic number of the element is called the effective atomic number of the substance [25]. This study found that the effective atomic number of patients in the S1 group was significantly higher than that in the D0 group, and the difference was statistically significant (*P* < 0.05). This may be due to the difference of substances, such as fat, protein, and cytokines, contained in hepatic ascites and cancerous abdominal effusion.

In terms of compassion of different types of spectral curve, 3 cases (6%) of the 50 patients in the S1 group had an ascending spectral curve, 47 cases (94%) had a descending spectral curve, and 37 cases (88.1%) of the 42 patients in the D0 group had an ascending spectral curve, and there were 5 cases (11.9%) of descending type. This indicated that the decreasing curve of hepatic ascites was dominant, while the increasing curve of cancerous peritoneal effusion was dominant. In addition, the slope of the spectral curve in the S1 group was significantly lower than that in the D0 group, and the difference was statistically significant (*P* < 0.05), suggesting that the slope of the spectral curve can be used to quantitatively evaluate the difference of the spectral curve in hepatic ascites and cancerous peritoneal effusion. It was believed that the difference in the spectral curve of peritoneal fluid between the two groups was mainly related to the difference of cells and components contained in the two groups. By calculating the diagnostic efficacy of some parameters in CT images on hepatic ascites, the sensitivity and specificity of water (iodine) were 0.927 and 0.836, respectively; the sensitivity and specificity of water (calcium) were 0.863 and 0.887, respectively, indicating that the CT parameters of water (iodine) and water (calcium) had good performance in diagnosing hepatic ascites, and the combined diagnosis of the two can be used clinically to diagnose hepatic ascites.

## 5. Conclusion

In this study, the AIHT algorithm for CT image reconstruction was proposed, and its performance was compared with that of previous algorithms. Then, 100 patients diagnosed with peritoneal effusion were selected as the research subjects, and 8 cases were excluded. The remaining was divided into 50 cases of the S1 group (hepatic ascites) and 42 cases of the D0 group (cancerous peritoneal effusion). Gemstone energy spectrum CT scanning was performed on all patients, and CT image parameters of the two groups were compared. The results showed that the AIHT-based CT image can better display the distribution of hepatic acids, and its parameters of CT value, effective atomic number, water (iodine), water (calcium), and spectral curve can help to identify hepatic acids, and especially water (iodine) and water (calcium) had high diagnostic performance. In conclusion, gem spectral CT has positive significance for the diagnosis of peritoneal effusion with cirrhosis and can be used as an effective method to examine, diagnose, and treat peritoneal effusion with cirrhosis. However, some limitations in the study should be noted. The sample size is small, which will reduce the power of the study. In the follow-up, an expanded sample size is necessary to strengthen the findings of the study.

## Figures and Tables

**Figure 1:** The processing results of CT images in the scanning range [0,90] by different algorithms. (a) RMSE of CT images in the scanning range [0,90]. (b) PSNR of CT images in the scanning range [0,90]. (c) The original image and the reconstructed image. ∗ represented statistically significant differences compared with AIHT algorithm (*P* < 0.05).

**Figure 2:** The processing results of CT images in scan range [0,120] by different algorithms. (a) RMSE of CT images in the scanning range [0,120]. (b) PSNR of CT images in the scanning range [0,120]. (c) The original image and the reconstructed image. ∗ represented statistically significant differences compared with AIHT algorithm (*P* < 0.05).

**Figure 3:** The age and sex ratio in the two groups. (a) Age and number of males and females. (b) Course of disease and BMI. (c) Diabetes, hypertension, and smoking.

**Figure 4:** CT image of cirrhotic effusion in a 48-year-old male patient. (a) and (b) were plain CT images; (c) and (d) were enhanced CT images. Red arrow marked ascites.

**Figure 5:** CT image of peritoneal effusion in a 53-year-old male patient with gastric cancer. (a) and (b) were plain CT images; (c) and (d) were enhanced CT images.

**Figure 6:** CT values of the two groups. (a) CT value under mixed energy. (b) CT value under single energy. ^∗^Compared with the S1 group, *P* < 0.05.

**Figure 7:** Comparison of paired basal substance concentration and effective atomic number between the two groups. (a) Water (calcium) concentration value and water (iodine) concentration value. (b) The effective atomic number. ^∗^Compared with the S1 group, *P* < 0.05.

**Figure 8:** Comparison of the spectral curve between the two groups. (a) The slope of spectral curve. (b) The spectral curve type of patients in group S1. (c) The spectral curve type of patients in group D0. ^∗^Compared with the S1 group, *P* < 0.05.

**Figure 9:** Diagnostic efficacy of some parameters in CT images on hepatic ascites.

## Data Availability

The data used to support the findings of this study are available from the corresponding author upon request.
